# Effects of Thymosin *β*4 on Myocardial Apoptosis in Burned Rats

**DOI:** 10.1155/2022/2129629

**Published:** 2022-03-03

**Authors:** Xiaoming Wu, Shusong Li, Xinshu Feng, Hailing Wen, Xiangxi Meng, Kui Sun

**Affiliations:** Department of Burnand Plastic Surgery, Affiliated Hospital of Chengde Medical College, Chengde, Hebei 067000, China

## Abstract

The aim of this study was to investigate the effects of thymosin *β*4 on myocardial apoptosis following burns. Fifty healthy Sprague Dawley (SD) rats were randomly divided into the normal control group, resuscitation group the low-dose T*β*4 (thymosin *β*4) group (2g), the medium-dose T*β*4 group (6g), and the high-dose T*β*4 group (18g). The rats were immersed in 95°C hot water for 18 seconds, and then the model of 30% body surface area (TBSA) III° scald was established. The resuscated rats were injected with lactate Ringer's solution for antishock rehydration, while the T*β*4 treatment group was injected with lactate Ringer's solution for antishock rehydration, and the animals were sacrificed 6 h after scald. The degree of histopathological damage was observed by HE (hematoxylin and eosin) staining. Western blot was used to detect STAT1 and STAT3 protein expression levels. Real-time PCR was used to detect mRNA expressions of STAT1 and STAT3. The results showed that the apoptosis rate of the resuscitation group was significantly higher than that of the control group (*P* < 0.01). Compared with the resuscitation group, the apoptosis rate of thymosin *β*4 in the treatment group was significantly reduced (*P* < 0.01). Compared with the normal control group, the expression of STAT1 protein was increased and the expression of STAT3 protein was decreased in model group rats after ischemia and reperfusion. Compared with the model group, the expression of STAT1 protein decreased and the expression of STAT3 protein increased after ischemia-reperfusion in the thymosin *β*4 treatment group. Thymosin *β*4 may protect the myocardium by downregulating STAT1 and upregulating STAT3 expression and inhibiting myocardial apoptosis induced by ischemia and reperfusion after severe scald injury.

## 1. Introduction

Early ischemia-reperfusion injury after a severe burn is one of the pathological bases of myocardial cell damage after burn, which can lead to cardiac dysfunction, induce or promote the aggravation of burn shock, and is often accompanied by myocardial cell apoptosis and tissue necrosis. Excessive myocardial cell apoptosis plays an important role in myocardial ischemia-reperfusion injury. Therefore, it is of great significance to effectively inhibit the excessive apoptosis of cardiomyocytes in the early stage of burn for maintaining cardiac function and promoting the recovery of cardiomyocytes. T*β*4, as a multifunctional peptide, is widely distributed in the body and plays an important role in promoting wound and corneal injury healing, myocardial cell repair, tissue regeneration, angiogenesis, antiapoptosis, and anti-inflammation [1]. Recent studies have suggested that T*β*4 has a neuroprotective effect and can reduce astrosporin-induced motor neuron death [2]. It can reduce the damage of excitatory amino acids to cortical neurons and the whole rat model [3] and improve the neurological injury symptoms of cerebral ischemia rats [4]. Deep second-degree burn can cause tissue cell damage and skin defense dysfunction, which may be related to the initiation of apoptosis [5]. The purpose of this study was to investigate the protective effect of adenomycin *β*4 on myocardial ischemia-reperfusion injury in rats. We established a rat model of severe scald to investigate the effects of thymosin *β*4 with different doses in the treatment of severe scalding and inhibited apoptosis after ischemia-reperfusion by downregulating STAT1 and upregulating STAT3 expression in myocardial cells. The study aims to provide an experimental basis for the early protection of clinical cardiomyocytes.

## 2. Materials and Methods

### 2.1. Ethical Approval

Research experiments conducted in this article with animals were approved by the Ethics Committee of Affiliated Hospital of Chengde Medical College and follow all guidelines, regulations, legal, and ethical standards as required for animals.

### 2.2. Main Reagents, Drugs, and Instrument

Thymosin *β*4 was provided by Baoding Shitao Import and Export Trading Co., Ltd. (Batch no.: T860463), an AnnexinV FITC Apoptosis Kit was purchased from Nanjing Kaiji Biotechnology Co., Ltd., flow cytometer (FACSCalibur flow cytometer) was purchased from BD Company, USA, and the rest reagents were all domestic pure products for analysis.

### 2.3. Experimental Animals and Grouping

A total of 50 healthy SD rats were purchased from Beijing Vital River Laboratory Animal Technology Co., Ltd. Twenty-five females and males were each selected and randomly divided into 5 groups: a sham burn group (control group), a resuscitation group, a *β*4 low-dose group (2 *μ*g), a T*β*4 medium-dose group (6 *μ*g), and a T*β*4 high-dose group (18 *μ*g). There were 10 rats in each group. The control group was immersed in a 37°C water bath for 18 s after scalding, the resuscitation group was intraperitoneally injected with Ringer's lactate solution (4 ml/% TBSA/kg) immediately after scalding, and the treatment group was injected with 2 *μ*g, 6 *μ*g, and 18 *μ*g of T*β*4 solution in the peritoneal cavity of rats, respectively, at the same time. Six hours after scalding, the rats were sacrificed and the myocardial tissue was collected for analysis.

### 2.4. Preparation of Animal Models

An intraperitoneal injection of 2% sodium pentobarbital (30 mg/kg) was used for anesthesia, followed by hair removal with 10% sodium sulfide. After 24 h, a water bath at 95°C for 18 s resulted in 30% TBSAIII° scald.

### 2.5. Routine Pathomorphological Observation of Myocardial Tissue

The myocardial tissue was embedded in paraffin. Three slices of 5 *μ*m were cut continuously at 1 mm intervals along the axis of the heart in the middle of the myocardium. The dewaxed sections of myocardial tissue were fixed on poly-L-lysine-coated slides. The tissue sections were dewaxed by xylene and gradient ethanol and stained with hematoxylin (Beyotime, Shanghai) for 3 min. It was differentiated with 1% ethyl alcohol hydrochloride for 30 s, then dyed with 0.5% eosin for 3 min, and then dehydrated and transparent with gradient ethanol and xylene successively. After drying in a fume hood, the sheet was sealed with neutral gum. The degree of myocardial injury in each group was observed under a microscope (Nikon, Japan).

### 2.6. Western Blot

The expression of STAT1 protein and STAT3 protein in cardiomyocytes was detected by western blot. The adherent cells were moistened and washed twice with PBS (phosphate-buffered saline) solution at 4°C, and the cell lysate precooled (Thermo, USA) by ice was added to extract the total protein of the cells. The protein was quantified by the BCA (Sigma USA) method. 90 *μ*g protein samples were collected, separated by 8% polyacrylamide gel electrophoresis, and transferred to polyvinylidene fluoride (PVDF) membrane. After blocking with 5% skimmed milk powder for 2 h, the primary antibody of rabbit anti-rat STAT1 and anti-rat STAT3 (Abcam, USA) diluted with 1 : 200 was incubated overnight at 4°C, and the secondary antibody diluted with 1 : 5 000 (Abcam, USA) was incubated at room temperature for 1 h. After washing with the membrane solution, color was developed with a chemiluminescence reagent (ECL), and the X-ray film was exposed, developed, and fixed. *β*-Actin (1 : 200 dilution) was used as an internal reference. The film is scanned by a scanner to obtain an image. The experiment was repeated 5 times in each group. The grayscale ratio of target protein bands to *β*-actin was calculated, and the relative expression levels of STAT1 and STAT3 proteins were calculated.

### 2.7. Flow Cytometry

The myocardium cells of each group were inoculated in a 6-well plate and prepared into single cell suspension with 0.125% trypsin digestive solution. The supernatant was discarded after centrifugation at 1000 r/min for 10 min. The supernatant was discarded and a 200 *μ*l binding buffer was added. Annexin-V/FITC (10 *μ*L) and 5 *μ*L FITC (KeyGEN BioTECH, Jiangsu) were mixed gently and reacted at room temperature for 15 min without light. A FACSCalibur flow cell analyzer was used to detect the apoptosis rate.

### 2.8. RT-PCR

The mRNA expression of STAT1 and STAT3 genes in cardiomyocytes was detected. Cells were collected and total RNA was extracted with TRIZOL. The extracted RNA samples were dissolved in water without RNase contamination. The absorbance values at 260/280 nm were determined using a universal RT-PCR kit (Solarbio, Beijing). The upstream primer sequence of the STAT1 gene was 5′ ATTATTGACGGGTTGTTTATGG 3′, the downstream primer sequence was 5′ GGTGCCTGTAGT CCTGGATG 3′, and the amplified product was 430 bp. The upstream primer sequence of the STAT3 gene was 5′CTGGCCGGAACAAGAGTG3′, the downstream primer sequence was 5′ GTGGATGCAAGGGTGGTG 3′, and the amplified product was 373 bp. The upstream primers of *β*-actin were 5′ CTGAGAGGGAAATCGTGCGT 3′ and the downstream primers were 5′TGGAAGGTGGACAGTGAGGC3′, and the amplified product was 448 bp. The amplified products were separated by electrophoresis with 2% agarose and then photographed by a UVP imaging analysis system. Quantity One software was used for grayscale analysis. Each experiment was repeated 5 times, and the grayscale ratio between target gene bands and *β*-actin was calculated.

### 2.9. Statistical Analysis

The experimental data were expressed in the form of *x* ± *s*. SPSS11.5 statistical software was used for statistical processing. One-way ANOVA was used for the comparison of measurement data between multiple groups, and *t*-test was used for pairwise comparison. *P* < 0.05 indicated a statistically significant difference. Each experiment was repeated three times.

## 3. Results and Discussion

### 3.1. Morphological Observation of Myocardium

The myocardial cells of rats in the control group were neatly arranged without inflammatory cell infiltration (Figure 1(a)). In the resuscitation group, the transverse lines of the myocardium were blurred or disappeared, the degree of myocardial cell swelling was obvious, the cell body was obviously enlarged, and part of the nucleus and cytoplasm disappeared. There was a large inflammatory cell infiltration (Figure 1(b)). In the thymosin *β*4 low-dose group (Figure 1(c)), the thymosin *β*4 medium-dose group (Figure 1(d)), and the thymosin *β*4 high-dose group (Figure 1(e)), the myocyte edema was reduced, the volume was significantly reduced, the nucleus was condensed, a few inflammatory cells were infiltrated, and a large number of normal myocytes were still present. The results indicated that thymosin *β*4 could significantly reduce the degree of myocardial histopathological injury after scalding in rats.

### 3.2. The Effect of Thymosin *β*4 on STAT1 and STAT3 Protein Expressions in Cardiomyocytes

Western blot results in Figure 2 showed that the ratio of STAT1 to its corresponding *β*-actin bands in the normal control group was 0.531 ± 0.006. Compared with the normal control group, the ratio of STAT1 to *β*-actin bands in the resuscitated group was 0.946 ± 0.007, which was significantly higher than that in the normal control group (*P* < 0.01). Compared with the resuscitation group, the ratio of STAT1 to its corresponding *β*-actin bands was 0.932 ± 0.005, 0.923 ± 0.004, and 0.596 ± 0.008, respectively. The expression of STAT1 protein in cardiomyocytes of rats treated with adenomycin *β*4 was significantly decreased (*P* < 0.05; *P* < 0.01). The ratio of STAT3 to *β*-actin bands in the normal control group was 0.751 ± 0.006. Compared with the normal control group, the ratio of STAT3 to *β*-actin bands in the resuscitation group was 0.432 ± 0.021, which was significantly lower than that in the normal control group (*P* < 0.01). Compared with the resuscitation group, the ratio of STAT3 to its corresponding *β*-actin bands was 0.474 ± 0.010, 0.566 ± 0.005, and 0.596 ± 0.008, respectively. The expression of STAT3 protein in cardiomyocytes of rats treated with adenomycin *β*4 increased significantly (*P* < 0.05; *P* < 0.01) (Table 1).

### 3.3. Detection of Cardiomyocyte Apoptosis

As shown in Figure 3, compared with the control group, the apoptosis rate in the resuscitation group was significantly increased (*P* < 0.01). Compared with the resuscitation group, the apoptosis rate of the thymosin *β*4 treatment group was decreased significantly (*P* < 0.05, *P* < 0.01, and *P* < 0.001), suggesting that thymosin *β*4 can reduce the apoptosis of rat cardiomyocytes caused by scalding.

### 3.4. The Effect of Thymosin *β*4 on the STAT1 mRNA Expression in Cardiomyocytes

As shown in Figure 4, the ratio of STAT1 to *β*-actin mRNA bands in the normal control group was 0.531 ± 0.006. Compared with the normal control group, the ratio of STAT1 mRNA bands to *β*-actin mRNA bands in the resuscitation group was 0.946 ± 0.007, which was significantly higher than that in the normal control group (*P* < 0.01). The ratio of STAT1 to *β*-actin mRNA bands in the thymosin *β*4 treatment group was 0.932 ± 0.005, 0.923 ± 0.004, and 0.596 ± 0.008. Compared with the resuscitation group, the ratio of STAT1 to *β*-actin mRNA bands decreased significantly (*P* < 0.05, *P* < 0.01, and *P* < 0.01).

### 3.5. The Effect of Thymosin *β*4 on the STAT3 mRNA Expression in Cardiomyocytes

As shown in Figure 5, the ratio of STAT3 mRNA bands to *β*-actin mRNA bands in the normal control group was 0.751 ± 0.006. Compared with the normal control group, the density of STAT3 mRNA bands decreased in the resuscitation group and the ratio of the gray level of *β*-actin mRNA bands in the resuscitation group was 0.432 ± 0.021. It is significantly lower than that in the normal control group (*P* < 0.01). The ratio of STAT3 to *β*-actin mRNA bands in the thymosin *β*4 treatment group was 0.474 ± 0.010, 0.566 ± 0.005, and 0.596 ± 0.0008, respectively, which were significantly increased compared with those in the resuscitation group (*P* < 0.05, *P* < 0.01, *P* < 0.01, and *P* < 0.01).

## 4. Discussion

In this study, animal modeling showed that thymosin *β*4 treatment improved severe scald to varying degrees, suggesting the value of thymosin *β*4 in the adjuvant treatment of scalding. In the pathogenesis of ischemia-reperfusion injury, apoptosis of myocardial tissue cells plays an important role in the pathological process of ischemia-reperfusion injury, that is to say, ischemia-reperfusion injury is realized by regulating the apoptotic process of myocardial tissue cells [6]. The decrease of cardiac function in the early burn is closely related to myocardial cell apoptosis. Therefore, inhibiting myocardial cell apoptosis can improve cardiac insufficiency [7, 8]. The results of this study indicated that apoptosis of cardiomyocytes occurred in rats after severe scalding, and adenothymidin *β*4 could inhibit the apoptosis of cardiomyocytes after severe scalding. It has been reported that thymosin *β*4 therapy is effective in the treatment of burn patients, especially those with early thymosin *β*4 intervention or high wound basement membrane tissue integrity [9, 10]. In this experiment, hematoxylin-eosin staining was used to observe the pathological damage degree of myocardial tissue of scald rats under the microscope. Compared with the control group, the swelling degree of myocardial cells in the resuscitation group was obvious, and the cell body was significantly enlarged. The volume of myocardium cells in groups with different doses of thymosin *β*4 was significantly reduced, the nucleus was condensed, a few inflammatory cells were infiltrated, and a large number of normal myocardium cells still existed. The results showed that thymosin *β*4 could significantly reduce the pathological damage of myocardium in scald rats.

The JAK2/STAT3 signaling pathway is involved in the expression of a large number of cytokines, growth factors, and hormones and also plays a crucial role in protecting the myocardium from an ischemia-reperfusion injury [11]. When it is inhibited, it can activate Caspase-3 and initiate apoptosis [12]. Studies have shown that the protective mechanism of decreasing myocardial cell apoptosis induced by ischemia-reperfusion in rats may be related to the regulation of the JAK2/STAT3 signaling pathway [13]. The activation of JAK2 can reduce STAT1 expression and increase the STAT3 expression, thereby inducing cell protection in the heart [14]. In the study of isolated rat cardiac cardiomyocytes, it was found that the phosphorylation induction of JAK2 and STAT3 in cardiac cardiomyocytes can protect the heart during perfusion [15]. Stephanou et al. [16] found that ischemia-reperfusion induced rapid phosphorylation of STAT1 instead of STAT3 in cardiomyocytes and that STAT1-transfected cardiomyocytes resulted in increased apoptosis after simulated ischemia, while STAT3-transfected cardiomyocytes reduced ischemia-induced apoptosis. It has been confirmed that a T*β*4 therapy can alleviate the neurological deficits in rats [17]. T*β*4 inhibits apoptosis and plays a neuroprotective role [18]. In this study, western blot was used to detect the effects of adenomycin *β*4 on the expression of STAT1 and 3 proteins in cardiomyocytes during ischemia and reperfusion. The results showed that compared with the normal control group, the expression of STAT1 protein was increased and the expression of STAT3 protein was decreased in model group rats after ischemia and reperfusion. Compared with the model group, the expression of STAT1 protein decreased and the expression of STAT3 protein increased after ischemia-reperfusion in the adenomycin *β*4 treatment group, which was consistent with studies by Stephanou et al. Therefore, it is of great significance to effectively inhibit the excessive apoptosis of myocardial cells in the early stage of burn for maintaining the power of heart pump and promoting the recovery of cardiac function.

As a multifunctional peptide, thymosin *β*4 (T*β*4) can specifically bind to G-actin and regulate actin polymerization. T*β*4 can promote wound tissue healing, myocardial repair, angiogenesis, antiapoptosis, and anti-inflammation. Kupatt et al. [19] topically applied adenothymidin *β*4 to enhance the antiacute myocardial ischemia-reperfusion injury effect of embryonic endothelial progenitor cells. Hinkel et al. [20] also reported that the local application of adenothymidin *β*4 can promote the protective effect of embryonic EPCs on the heart. Compared with the control group, the apoptosis rate in the resuscitation group was significantly increased (*P* < 0.01). Compared with the resuscitation group, the apoptosis rate of the thymosin *β*4 treatment group was decreased significantly (*P* < 0.05; *P* < 0.01), suggesting that thymosin *β*4 can reduce the apoptosis of rat cardiomyocytes caused by a scald injury. The results of this study indicated that apoptosis of cardiomyocytes occurred in rats after severe scalding, and adenothymidin *β*4 could inhibit the apoptosis of cardiomyocytes after severe scalding.

The purpose of this study was to investigate the protective effect of adenomycin *β*4 on myocardial ischemia-reperfusion injury in rats and to investigate the effect of adenomycin *β*4 on myocardial cells after scalding in SD rats and its molecular mechanism at the cellular level. In this study, RT-PCR was used to detect the effects of adenothymidin *β*4 on STAT1 and STAT3 mRNA expressions in myocardial cells after ischemia-reperfusion after severe scalding in rats. The results showed that the expression of STAT1 mRNA in myocardial cells in the resuscitation group was increased after ischemia-reperfusion compared with the normal control group. The STAT3 mRNA expression decreased. Compared with the resuscitation group, the expression of STAT1 mRNA was decreased and the expression of STAT3 mRNA was increased in cardiomyocytes in the treated group after ischemia-reperfusion, suggesting that the expression of STAT1 mRNA in cardiomyocytes was decreased in the treated group, suggesting that the expression of STAT3 mRNA was decreased in the treated group after ischemia-reperfusion. The results of this study suggest that T*β*4 has a potential clinical value in the treatment of scald. However, this study was only discussed at the level of animal model. In addition, the dose, concentration, and timing of administration need to be further demonstrated, which is also the deficiency of this study.

## 5. Conclusion

The results of this study indicate that the apoptosis of myocardial cells occurs after severe scald ischemia-reperfusion in rats, and adenothymidin *β*4 inhibits the apoptosis of myocardial cells after severe scald. Thymosin *β*4 may protect the myocardium by downregulating STAT1 mRNA expression and upregulating STAT3 mRNA expression and inhibiting myocardial apoptosis induced by ischemia and reperfusion after severe scald injury. However, STAT regulates the expression of myocardial protective proteins through transcriptional translation, so as to participate in the protective effect of ischemia-reperfusion injury after severe scald.

## Figures and Tables

**Figure 1:** The degree of myocardial cell injury was detected by HE staining magnification of (×100). (a) Normal control group; (b) resuscitation group; (c) low-dose T*β*4 group (2g); (d) medium-dose T*β*4 group (6g); (e) high-dose T*β*4 group (18g). (c–e) The pathological damage of myocardial tissue in scald rats treated with T*β*4 in different doses.

**Figure 2:** The effect of thymosin *β*4 on p-STAT1 and P-STAT3 protein expression in rat cardiomyocytes after scald injury. (1) normal control group; (2) resuscitation group; (3) low-dose T*β*4 group (2g); (4) medium-dose T*β*4 group (6g); (5) high-dose T*β*4 group (18g). (a) Protein expression of STAT1 in cardiomyocytes of the resuscitation group and T*β*4 treatment group. (b) Protein expression of STAT3 in cardiomyocytes of the resuscitation group and T*β*4 treatment group.

**Figure 3:** Effects of different doses of thymosin *β*4 on myocardial apoptosis induced by scald. (a) Normal control group; (b) resuscitation group; (c) low-dose T*β*4 group (2g); (d) medium-dose T*β*4 group (6g); (e) high-dose T*β*4 group (18g).

**Figure 4:** The effect of thymosin *β*4 on STAT1 mRNA expression in cardiomyocytes. The mRNA of STAT1 in myocardial tissue of scald rats was determined by RT-PCR. ^*∗∗∗*^*P* < 0.001, the difference was statistically significant compared with normal control group; ^Δ^*P* < 0.05, ^ΔΔ^*P* < 0.01, and ^ΔΔΔ^*P* < 0.001, the resuscitation group was significantly different from the resuscitation group.

**Figure 5:** The effect of thymosin *β*4 on STAT3 mRNA expression in cardiomyocytes. The mRNA of STAT3 in myocardial tissue of scald rats was determined by RT-PCR. ^*∗∗∗*^*P* < 0.001, the difference was statistically significant compared with normal control group; ^Δ^*P* < 0.05, ^ΔΔ^*P* < 0.01, and ^ΔΔΔ^*P* < 0.001, the resuscitation group was significantly different from the resuscitation group.

**Table 1:** The effect of thymosin *β*4 on STAT1 and STAT3 protein expressions in rat myocardial tissue after scald injury.

Group	Degree (*μ*g/L)	P-STAT1/*β*-actin	P-STAT3/*β*-actin
Normal control group	—	0.531 ± 0.006	0.751 ± 0.006
Resuscitation group	—	0.946 ± 0.007^*∗*^	0.432 ± 0.021^*∗*^
Low-dose T*β*4 group (2g)	2	0.932 ± 0.005^Δ^	0.474 ± 0.010^ΔΔ^
Medium-dose T*β*4 group (6g)	6	0.923 ± 0.004^ΔΔ^	0.566 ± 0.005^ΔΔΔ^
High-dose T*β*4 group (18g)	18	0.596 ± 0.008^ΔΔΔ^	0.596 ± 0.008^ΔΔΔ^

Western blot was used to determine the effects of thymosin *β*4 on the expression of STAT1 and STAT3 proteins in myocardium of scald rats. The data were the mean ± label difference (*X* ± *S*) of three independent experiments. *P* < 0.001^*∗*^ vs normal control group; *P* < 0.05^Δ^, *P* < 0.01^ΔΔ^, and *P* < 0.001^ΔΔΔ^ vs resuscitation group.

## Data Availability

The datasets used and/or analyzed during the current study are available from the corresponding author on reasonable request.
